The article "Influence of Nursing Intervention Based on Risk Assessment Model on Self-Efficacy and Postoperative Rehabilitation of Surgical Patients" was retracted in 2023. Reasons: suspected computer-generated content; unreliable results or conclusions; concerns about the data; concerns about the results or conclusions.

# Influence of Nursing Intervention Based on Risk Assessment Model on Self-Efficacy and Postoperative Rehabilitation of Surgical Patients

**DOI:** 10.1155/2022/6750320

**Published:** 2022-04-13

**Authors:** Yanfang Yang, Peng Chen, Cuili Jiao

**Affiliations:** Department of Anesthesiology, Cangzhou Central Hospital, Cangzhou, Hebei, China

## Abstract

The study aims to explore the effect of nursing intervention based on risk assessment model on self-efficacy and postoperative rehabilitation of surgical patients. The study applied a risk assessment model to the behavioral intervention of rehabilitation exercise in patients after percutaneous coronary intervention (PCI). A total of 157 patients were selected from a certain hospital, with 52 cases in the experimental group and 55 cases in the control group. A comprehensive cardiac rehabilitation intervention strategy based on TTM is given by researchers trained with professional knowledge, including dividing the stages of behavior change, developing a rehabilitation exercise plan through exercise teaching and exercise training, diet and lifestyle guidance, and urging patients to take regular medication and regular follow-up. The stage of rehabilitation movement behavior change improved. The preexperiment health status was (35.39 ± 14.31), and the overall health of the control group was (32.59 ± 15.41). Overall health status and QOL scores were relatively low in both the groups. The intervention group scored higher than the control group. After coronary stent implantation, the heart restores its original pumping function, various organs and tissues receive effective blood perfusion, and the symptoms of myocardial infarction such as profuse sweating, dizziness, fatigue, and precordial discomfort are effectively relieved. The physical discomfort can gradually improve or even recover to the functional state before the onset of the disease. Before the intervention, the self-efficacy score of the intervention group was (23.68 ± 4.49). After the intervention, the self-efficacy score of the intervention group was (26.21 ± 4.09), while the self-efficacy score of the control group before the intervention was (22.21 ± 4.1). After the intervention, the self-efficacy score of the control group was (25.23 ± 4.41). Although the self-efficacy score of the control group was improved, the difference was small, and the intervention effect was not obvious. It indicates that risk assessment intervention can improve patients' self-efficacy level and quality of life of postoperative rehabilitation patients.

## 1. Introduction

Nursing intervention based on self-efficacy refers to improving the subjective judgment of patients through a variety of nursing methods so that patients can eliminate their fear of disease, increase their recognition of their own abilities, increase patients' belief in their ability to overcome the disease, gain health, and boost confidence in disease treatment and prognosis, thereby eliminating bad psychology, improving compliance with treatment and nursing, and ultimately improving the quality of life of patients. Once coronary artery spasm or stenosis lead to blood interruption, severe and persistent acute ischemia of the corresponding myocardium can occur, leading to the onset of acute myocardial infarction and the decrease of life quality [1, 2]. Studies have shown that regular rehabilitation exercise can improve vascular endothelial elasticity, reduce controllable risk factors for coronary heart disease, delay disease progression, improve cardiac functional reserve, increase cardiac output, and improve quality of life [3]. The compliance of patients with rehabilitation exercise after PCI directly affects the quality of life and long-term prognosis of patients. It is particularly important to carry out effective behavioral intervention to improve the compliance of rehabilitation exercise. In this study, a risk assessment model is used in the behavioral intervention of rehabilitation exercise in patients after PCI.  Figure 1 presents a general framework for information risk assessment [4].

The article "Influence of Nursing Intervention Based on Risk Assessment Model on Self-Efficacy and Postoperative Rehabilitation of Surgical Patients" was retracted in 2023. Reasons: suspected computer-generated content; unreliable results or conclusions; concerns about the data; concerns about the results or conclusions.

## 2. Literature Review

In response to this research question, Saboula et al. proposed that the comprehensive assessment of the elderly has an important guiding role and clinical application value for the midterm care after acute onset and subacute stage of chronic diseases in the elderly [5]. Paynter et al. explored the midterm care model for elderly patients with acute exacerbation of chronic obstructive pulmonary disease, and clarified the entry and exit criteria, team composition, personnel responsibilities, and patient circulation for elderly patients with chronic obstructive pulmonary disease. The process and implementation plan provide a strong basis and reference for other midterm care models, processes, and implementation of acute exacerbation of chronic diseases in the elderly [6]. Foley et al. investigated the awareness of midterm care of fracture patients and found that fracture patients' awareness of midterm care is generally insufficient, and it tends to weaken with age; a survey of midterm care needs for fracture patients shows that rehabilitation guidance, condition observation, medication guidance, health education, and wound care are technologies that require high midterm care for fracture patients [7]. Birns and Bhalla provided discharge guidance and positive nursing intervention outside the hospital for patients after coronary stent placement, which significantly improved the patient's self-management ability and quality of life [8]. Khalife-Zadeh et al. believed that it is very necessary to change the bad lifestyle through postoperative health education for patients and prevent the development of heart disease after PCI [9]. The results of Weingart et al.'s study showed that continuous care for patients after CABG can promote the recovery of cardiac function, help patients improve their lifestyle, reduce the occurrence of major adverse cardiac events (MACE), and reduce hospital readmissions risk [10]. In the study of Moeini et al., 110 patients after CABG underwent home walking rehabilitation training four times a week for five consecutive weeks, after 2 months of out-of-hospital rehabilitation nursing intervention [11]. Salehi et al.'s study showed that the quality of life of discharged patients was significantly improved after 1 year of hospital–community–family diversified cardiac rehabilitation consisting of community nurses, general practitioners, and in-hospital medical staff [12]. The study by Phuyal and Pottle showed that continuous rehabilitation nursing can provide patients with knowledge related to cardiac rehabilitation after CABG and methods for postoperative pain relief [13]. Ashur et al. believed that psychological intervention methods include self-relaxation, self-regulation, among others, and lifestyle interventions include instructing patients to perform respiratory function training, performing rehabilitation exercises in stages, guiding medication according to patients' conditions, and guiding dietary nutrition, etc. [14]. A comprehensive cardiac rehabilitation intervention strategy based on TTM is given by researchers trained with professional knowledge, including dividing behavioral change stages, developing rehabilitation exercise plans through exercise teaching and exercise training, diet and lifestyle guidance, and urging patients to take regular medication and regular follow-up. Feasible rehabilitation exercise programs are provided for patients so that they can have methods to follow, solve their needs, support their thoughts, so as to enhance their confidence and determination to carry out rehabilitation exercises. The patient's self-efficacy has been significantly improved, mainly because the researchers used the self-re-evaluation and awakening mechanism to effectively stimulate the patient's motivation to participate in cardiac rehabilitation, make the patient change from passive to active, and improve disease self-management and disease control ability. It shows that the behavioral intervention based on the risk assessment model can promote the physical and psychological recovery of the patients after surgery, improve the patients' self-emotional management, and the ability to cope with the disease, and promote the psychological health of the patients after coronary stent implantation.

The article "Influence of Nursing Intervention Based on Risk Assessment Model on Self-Efficacy and Postoperative Rehabilitation of Surgical Patients" was retracted in 2023. Reasons: suspected computer-generated content; unreliable results or conclusions; concerns about the data; concerns about the results or conclusions.

## 3. Method

### 3.1. Research Object

#### 3.1.1. Inclusion Criteria

Age: 40–70 years old; confirmed by coronary angiography and successfully performed stent implantation; good understanding and communication skills [15].

#### 3.1.2. Exclusion Criteria

Those with cognitive impairment or with mental illness who cannot cooperate; with severe heart failure or hemodynamic instability with serious complications; or other physical diseases. Patients who dropped out due to various reasons; all enrolled patients signed the informed consent.

#### 3.1.3. Grouping Method

The control group was admitted to the third treatment area on the fifth floor of the Department of Cardiology, while the intervention group was admitted to the third treatment area on the fourth floor of the Department of Cardiology.

### 3.2. Research Methods

#### 3.2.1. Preexperiment

Through 12 pretests, some controllable factors that may disturb the effect of the experimental observation were found, and corrections and changes were made in a timely manner: the intervention time was adjusted to minimize the time for disturbing the patient's rest and treatment. After the patients are discharged from the hospital, close contact is kept with the patients and their families, continuously understanding the dynamics of the patients outside the hospital.

#### 3.2.2. Data Collection Method

The selected 107 patients after PCI, completed the behavior change stage questionnaire, general self-efficacy scale (GSES), and short form 36 questionnaire (SF-36) on the second day after the operation. Blood samples were collected, blood pressure was measured, and general information, baseline behavior changes, quality of life, and self-efficacy levels of patients after PCI were evaluated, blood pressure and blood lipid levels were recorded, and the original data of the research subjects were established.

After the evaluation, the control group received routine nursing care, life nursing, and health education during hospitalization, and a weekly telephone follow-up within 1 month after discharge, and once a month after 1 month for 6 months (nine times in total). The patients were urged to review and conduct routine enquiries. After 1 month, monthly telephone follow-up was conducted once for 6 months (nine times in total) to dynamically understand the transition stage of patients' healthy behavior and the implementation of the rehabilitation exercise plan, and timely adjust the intervention strategy and exercise prescription according to the patients' feedback. Six months after discharge, the two groups of patients filled out the above questionnaire again, collected blood samples, measured blood pressure, and compared the health behavior, quality of life, and self-efficacy [16].

The article "Influence of Nursing Intervention Based on Risk Assessment Model on Self-Efficacy and Postoperative Rehabilitation of Surgical Patients" was retracted in 2023. Reasons: suspected computer-generated content; unreliable results or conclusions; concerns about the data; concerns about the results or conclusions.

#### 3.2.3. Research Tools

The quality of life of patients was measured using the SF-36 short form of quality of life, which mainly included eight dimensions, including physiological function, physiological function, somatic pain, general health, energy, social function, emotional function, and mental health, with 24 items. The standardized score for each dimension ranges from 0 to 100, with higher scores indicating better quality of life for patients.

#### 3.2.4. Other Observation Index Measurement and Judgment Criteria

Judgment of rehabilitation exercise compliance: patients who reach 80% or more of the total recommended weekly exercise time are considered to have good compliance, and patients who reach 60% or more of the total weekly recommended exercise time are considered to have good compliance. Patients with a time of less than 60% were considered to be in poor compliance.

Blood pressure measurement method: After resting for 5 minutes in the morning, use a Mercury sphygmomanometer to measure the blood pressure of the brachial artery of the left upper arm in a sitting position (because the puncture site of the PCI operation is located in the radial artery of the right upper extremity, the blood pressure of the brachial artery of the left upper arm is selected) [17].

### 3.3. Intervention Method of Control Group

After the patients returned to the ward after surgery, they were given routine postoperative medication care and skin incision care at the puncture site. Postoperative education was given, and postoperative precautions and adverse reactions of anticoagulants were introduced. Postoperative hydration therapy was given, and pressure at the puncture site was given. The hemostat was periodically decompressed. It is necessary to observe whether there was bleeding and swelling on the skin at the puncture site, and whether there was a tendency to bleeding (whether the gums, nasal mucosa, and fundus were bleeding), instruct the patient to eat a low-salt, low-fat, light and easily digestible liquid diet, and instruct the patient to drink more water to promote the excretion of the contrast agent [18].

### 3.4. Intervention Method of Intervention Group

A comprehensive cardiac rehabilitation intervention strategy based on TTM is given by researchers trained with professional knowledge, including dividing behavioral change stages, developing rehabilitation exercise plans through exercise teaching and exercise training, diet and lifestyle guidance, and urging patients to take regular medication and regular follow-up [19].

The article "Influence of Nursing Intervention Based on Risk Assessment Model on Self-Efficacy and Postoperative Rehabilitation of Surgical Patients" was retracted in 2023. Reasons: suspected computer-generated content; unreliable results or conclusions; concerns about the data; concerns about the results or conclusions.

#### 3.4.1. Division of the Stages of Behavior Change

First, the researchers conducted a one-to-one assessment of the patients on the first postoperative day to assess the stage of change in the patients' behavior. According to the assessment results, cardiac rehabilitation interventions that match the stage of change are implemented for patients, once a day, 20 minutes each time, and given three to five times until discharge.

Preintentional stage: Use the strategies of consciousness arousal and vivid release in TTM to help patients recall their feelings since the illness in a timely manner. Through role analysis, it is recognized that there is irregular drug use, lack of rehabilitation exercise, and poor eating habits among the patients. Providing the knowledge of secondary prevention after coronary heart disease interventional therapy by playing audio-visual teaching materials and multimedia lectures, etc., makes them realize that the recurrence of stent thrombosis is often closely related to irregular physical exercise, and warns patients that if they do not perform cardiac rehabilitation exercises according to the doctor's orders after surgery, adverse consequences will be caused. It can help them look for intrinsic motivations for behavioral change.

Intentional stage: With the help of self-re-evaluation and environmental re-evaluation strategies in TTM, the internal and external factors that hinder patients from changing unhealthy behaviors and habits are analyzed encouraging them to overcome obstacles. A WeChat group is created to provide a platform for communication between patients. A patient in the maintenance phase is invited to share the benefits of long-term regular exercise every month, distribute a health handbook for safe exercise, and introduce the appropriate types of exercise, and number of times for patients after coronary stent implantation, encouraging them to overcome obstacles, and promoting the continuous transformation of patients to healthy behaviors [20].

Preparatory stage: Use the strategies of self-liberation and social liberation in TTM to discuss with patients the different problems that may arise in the process of behavioral change and assist and guide the patients to formulate a feasible cardiac rehabilitation exercise plan. Cardiac rehabilitation physicians set up a health education lecture hall, formulate a health education curriculum, and regularly hold “PCI-Heart Action” special lectures on cardiac rehabilitation knowledge once a week, 60 minutes each time. Introduce the precautions for activities after coronary stent implantation, and guide patients to learn to measure their own pulse, master the correct exercise method and amount of exercise, make patients understand the main role of the drugs they take, the observation and treatment of adverse reactions, and the prevention of emergency cardiovascular events and countermeasures.

The article "Influence of Nursing Intervention Based on Risk Assessment Model on Self-Efficacy and Postoperative Rehabilitation of Surgical Patients" was retracted in 2023. Reasons: suspected computer-generated content; unreliable results or conclusions; concerns about the data; concerns about the results or conclusions.

#### 3.4.2. Exercise Teaching

The researchers personally went to the ward to lead the patients to the rehabilitation treatment room for one-on-one rehabilitation exercise teaching, better at 2–4 p.m., three to five times a week, avoiding the patient's treatment time to improve the patient's participation rate.

#### 3.4.3. Assisting in the Formulation of Individualized Exercise Prescriptions

The actual situation of the patient must be comprehensively considered. A safe and feasible exercise prescription must be formulated with the patient in combination with factors such as age, disease progression, cardiopulmonary function, exercise habits, and psychological, social, and economic factors.

#### 3.4.4. Monitoring during Exercise

When starting rehabilitation training, it must be monitored by the researchers, so as not to cause any discomfort, as it is a normal response to increase the heart rate by 10–20 beats/min. When the heart rate increases <10 beats/min during exercise, the amount of exercise can be increased, and the trainee can be entered into the first stage of training. During exercise, if the heart rate increases by >20 beats/min, the systolic blood pressure decreases by more than 15 mmHg, and if arrhythmia occurs or the ECG ST segment, ischemia type decreases by >0.1 mV or increases by 20.2 mV, then it should return to the previous exercise level. When the heart rate changes more than 20 beats/min or the blood pressure changes more than 20 mmHg, the exercise process should be slowed down or stopped. To teach patients to measure their pulse by themselves, the highest heart rate (170—age) is generally used as the appropriate heart rate during exercise. After stopping the activity, the heart rate should return to normal within 3–5 min.

#### 3.4.5. Developing a Cardiac Rehabilitation Exercise Plan

The researchers worked out a feasible cardiac rehabilitation exercise plan with the patients in combination with the number of stents implanted and their daily life habits, including daily dietary guidance goals (blood pressure, blood lipid monitoring, and management), daily physical activity guidance (specific exercise and the level of work activity), daily stress emotional guidance, and discharge precautions. If the patient's behavioral change stage of participating in rehabilitation exercises is regressed, it is necessary to help him analyze the reasons, summarize experiences, and reformulate the intervention strategy, and then implement and reevaluate.

The article "Influence of Nursing Intervention Based on Risk Assessment Model on Self-Efficacy and Postoperative Rehabilitation of Surgical Patients" was retracted in 2023. Reasons: suspected computer-generated content; unreliable results or conclusions; concerns about the data; concerns about the results or conclusions.

#### 3.4.6. Regular Follow-Up

The patients were divided into three groups according to their discharge dates (patients discharged from the hospital on the 1st to 10th, 11th to 20th, and 20th to 30th of each month), and the corresponding groups were followed up by telephone every Friday to dynamically understand the behavior change stage of patients and the implementation of the cardiac rehabilitation exercise plan. The patients were followed up by telephone once a week within one month after discharge, changed to once a month after one month, and followed up for 6 months, a total of nine times. The patients' willingness to change behavior was continuously evaluated, and out-of-hospital rehabilitation exercise behavior monitoring was carried out using the self-designed and developed follow-up questionnaire after coronary stent implantation. The members of the research team regularly check and summarize the patients' rehabilitation exercise log and the completion of the goals once a week, give affirmation and encouragement to the patients who have completed the goals, carefully analyze the reasons for those who fail to achieve the goals, and timely assess the patients' compliance with rehabilitation exercise, give corresponding behavioral guidance, and adjust the intervention strategy and cardiac rehabilitation exercise plan in time according to the patient's feedback.

### 3.5. Statistical Methods

After the data was entered in Excel, SPSS 17.0 statistical software was used for analysis and processing, and the results were analyzed by statistical methods such as descriptive statistics, chi-square test, *t*-test, and rank sum test analysis; the test level was set to *a* = 0.05 for both sides.

1. Descriptive statistics: The general data of the surveyed subjects are carried out by frequency, percentage, mean, and standard deviation.
2. Two independent samples *t*-test, rank sum test, and chi-square test: the general data of the two groups were compared by the chi-square test, and the rank data was by the rank sum test; the quantitative data conforming to the normal distribution was tested by the two independent samples *t*-test.

## 4. Results and Analysis

### 4.1. Comparison of Behavior Change Stages before and after Intervention in Two Groups of Patients

As shown in Table 1, there were no special differences in the behavioral change stages of the two groups, and the postintervention behavior change stage of the rehabilitation movement was higher than that of the control group.

The article "Influence of Nursing Intervention Based on Risk Assessment Model on Self-Efficacy and Postoperative Rehabilitation of Surgical Patients" was retracted in 2023. Reasons: suspected computer-generated content; unreliable results or conclusions; concerns about the data; concerns about the results or conclusions.

### 4.2. Comparison of the Compliance of Rehabilitation Exercise between the Two Groups before and after Intervention (Figures 2 and 3)

### 4.3. Comparison of the Scores of Each Dimension of Quality of Life between the Two Groups before and after the Intervention

A comparison of the scores of each dimension of quality of life between the two groups of patients before intervention is shown in Table 2. A comparison of the scores of each dimension of quality of life between the two groups of patients after the intervention is shown in Table 3.

### 4.4. Comparison of General Self-Efficacy Scores between the Two Groups before and after Intervention

As shown in Figures 4 and 5, no overall self-performance scores between the first two groups of intervention varied significantly and higher overall self-performance scores in the intervention group than the control group, which were statistically significant. Overall self-efficiency scores after the intervention were statistically different when compared to the intervention group.

### 4.5. Comparison of Blood Pressure and Lipid Levels before and after Intervention

A comparison of blood pressure and blood lipid levels between the two patient groups before the intervention is shown in Table 4. A comparison of blood pressure and blood lipid levels in the two groups after the intervention is shown in Table 5.

### 4.6. Discussion

#### 4.6.1. The Effect of Nursing Intervention of Risk Assessment Model on the Quality of Life of Patients after PCI

Studies have shown that the designed intervention program has a significant effect on improving the quality of life of patients. The individualized exercise prescription and cardiac rehabilitation plan formulated by the researchers prepared for the rehabilitation exercise of patients after discharge and improved the willingness of patients to perform rehabilitation exercise after PCI. It has been recognized that cardiac rehabilitation can improve the functional reserve of patients after PCI. By increasing coronary blood supply, increasing vascular endothelial oxygen content, enhancing cell activity, and maintaining vascular patency, it can effectively reduce the risk of restenosis of diseased blood vessels and reduce the occurrence of ischemic adverse cardiovascular events in patients with coronary heart disease.

The results (Table 2) showed that before the intervention, the general health status of the intervention group was (35.39 ± 14.31) points, and the general health status of the patients in the control group was (32.59 ± 15.41) points. The reason for this analysis is that there are many middle-aged and elderly patients selected in this study, with low educational level, less access to health knowledge, lack of disease-related knowledge, failure to adopt healthy behavior habits and lifestyles, and most of these patients are accompanied by high blood pressure, diabetes. These predisposing factors are more likely to cause postoperative complications.

The article "Influence of Nursing Intervention Based on Risk Assessment Model on Self-Efficacy and Postoperative Rehabilitation of Surgical Patients" was retracted in 2023. Reasons: suspected computer-generated content; unreliable results or conclusions; concerns about the data; concerns about the results or conclusions.

The general health status scores of both the groups improved after the intervention (see Table 3). After coronary stent implantation, the heart restores its original pumping function, and various organs and tissues receive effective blood perfusion. Myocardial infarction symptoms such as profuse sweating, dizziness, fatigue, and precordial discomfort are effectively relieved, and the body discomfort can be gradually improved or even returned to functional status before the onset of disease. With the recovery of myocardial blood supply and improvement of cardiac function after coronary stenting, the pain in the precordial area is effectively relieved, and the patient's disease is effectively controlled. At the same time, the health education and follow-up work of the two groups of patients enabled the patients to come to the hospital for reexamination in a timely manner, early detection of abnormal changes in the cardiovascular system, and timely administration of drugs or surgical treatment, which prevented the occurrence of some adverse cardiovascular events.

#### 4.6.2. Influence of Nursing Intervention of Risk Assessment Model on Self-Efficacy of Patients after PCI

Clinical treatment methods focus too much on symptomatic treatment often ignoring the patient's self-feeling and the patient's mental illness. Patients with coronary heart disease are prone to bad emotions such as anxiety and depression due to repeated attacks and repeated hospitalizations, which can further aggravate the patient's condition.

## 5. Conclusion

This study proposes the effect of nursing intervention based on risk assessment model on the self-efficacy and postoperative rehabilitation of surgical patients and provides intervention treatment for patients diagnosed by coronary angiography. It can improve the subjective initiative of the patients, enable the patients to participate in the management of their own diseases, maintain a good emotional state, make them feel respected, and improve their disease coping ability. The improvement of mental and psychological state improves the patient's compliance with treatment and enables the implementation of the treatment plan. This article provides patients with a feasible rehabilitation exercise program so that patients can have a method to follow, meet the needs of the patients, support the patients' thoughts, so as to enhance their confidence and determination to perform rehabilitation exercises. The patient's self-efficacy has been significantly improved, mainly because the researchers used the self-re-evaluation and awakening mechanism to effectively stimulate the patient's motivation to participate in cardiac rehabilitation, make the patient change from passive to active, and improve the self-management of the disease and the ability to control the disease. It shows that the behavioral intervention based on the risk assessment model can promote the physical and psychological recovery of the patients after surgery, improve the patients' self-emotional management and the ability to cope with the disease, and promote the psychological health of the patients after coronary stent implantation. In the future, long-term (1–2 years) rehabilitation exercise behavior intervention based on cross-theoretical models will be implemented for patients after PCI, and the long-term quality of life, survival rate, and recurrence rate of patients will be tracked to further enrich the research content. The results of the study showed (see Figures 4 and 5) that the self-efficacy score of the intervention group was (23.68 ± 4.49) before the intervention, and the self-efficacy score of the intervention group after the intervention was (26.21 ± 4.09), and the difference was statistically significant before and after the intervention (*P* < 0.05), while the self-efficacy score of the control group before the intervention was (22.21 ± 4.1), and the self-efficacy score of the control group after the intervention was (25.23 ± 4.41). Although the self-efficacy score of the control group improved, the difference was small. The effect is not obvious. It suggests that risk assessment interventions can improve patients' self-efficacy levels [21].

The article "Influence of Nursing Intervention Based on Risk Assessment Model on Self-Efficacy and Postoperative Rehabilitation of Surgical Patients" was retracted in 2023. Reasons: suspected computer-generated content; unreliable results or conclusions; concerns about the data; concerns about the results or conclusions.

## Figures and Tables

**Figure 1:** Framework of information risk assessment.

**Figure 2:** Comparison of rehabilitation exercise compliance between the two groups before intervention.

**Figure 3:** Comparison of rehabilitation exercise compliance between the two groups after intervention.

**Figure 4:** A comparison of general self-efficacy between the two groups before intervention.

**Figure 5:** A comparison of general self-efficacy between the two groups after intervention.

**Table 1:** A comparison of behavior change stages before and after intervention in two groups of patients.

Stage of change	Before intervention		*Z*	*P*	After intervention		*Z*	*P*
	Intervention group	Control group			Intervention group	Control group		
Preintentional stage	18	20	0.139	0.879	1	16	5.861	<0.001
Intentional stage	21	21			3	9		
Preparation stage	10	9			5	16		
Action stage	4	5			42	16		
Maintenance stage	4	4			6	3		

**Table 2:** A comparison of scores of each dimension of quality of life between the two groups before intervention (*X* ± *S*).

Item	Intervention group	Control group
Physiological function	65.49 ± 20.67	65.35 ± 18.56
Physiological function	25.68 ± 9.61	22 65 ± 8.43
Body pain	55.19 ± 20.29	50.35 ± 18.42
General health	35.39 ± 14.31	32.59 ± 15.41
Energy	52.41 ± 20.29	58.45 ± 15.65
Social function	67.42 ± 26.28	70.12 ± 19.32
Emotional function	50.51 ± 42.01	43.65 ± 38.32
Mental health	52.43 ± 23.61	45.23 ± 19.42

**Table 3:** A comparison of various dimensions of quality of life between the two groups after intervention (*X* ± *S*).

Item	Intervention group	Control group
Physiological function	73.62 ± 16.79	66.28 ± 15.41
Physiological function	31.25 ± 10.11	30.58 ± 11.31
Body pain	68.56 ± 22.43	65.24 ± 20.62
General health	45.68 ± 18.42	36.58 ± 16.64
Energy	55.65 ± 22.71	62.561 ± 18.53
Social function	77.68 ± 25.64	74.23 ± 26.91
Emotional function	54.12 ± 40.23	46.34 ± 36.41
Mental health	57.25 ± 21.32	46.15 ± 22.56

**Table 4:** A comparison of blood pressure and blood lipid levels in the two groups before intervention (*X* ± *S*).

Item	Intervention group	Control group
SBP (mm Hg)	130.54 + 18.61	130.07 + 19.23
DBP (mm Hg)	80.17 + 12.41	75.89 + 13.64
TC (mmol/L)	4.77 + 0.79	4.83 + 0.94
TG (mmol/L)	2.10 + 1.11	2.07 + 1.13
HDL-C (mmol/L)	1.19 + 0.42	1.18 + 0.23
LDL-C (mmol/L)	2.83 + 0.68	2.94 + 0.691

**Table 5:** A comparison of blood pressure and blood lipid levels in the two groups after intervention (*X* ± *S*).

Item	Intervention group	Control group
SBP (mm Hg)	120.73 + 18.41	128.09 + 18.42
DBP (mm Hg)	78.48 + 11.88	74.69 + 11.32
TC (mmol/L)	4.17 + 0.72	4.52 + 0.87
TG (mmol/L)	1.36 + 0.71	2.00 + 0.59
HDL-C (mmol/L)	1.22 + 0.28	1.29 + 0.44
LDL-C (mmol/L)	2.68 + 0.63	2.85 + 0.59

## Data Availability

The data used to support the findings of this study are available from the corresponding author upon request.
